The article "MicroRNA-744-5p suppresses tumorigenesis and metastasis of osteosarcoma through the p38 mitogen-activated protein kinases pathway by targeting transforming growth factor-beta 1" was retracted in 2026. Reasons: concerns about the data; concerns about the results or conclusions.

# MicroRNA-744-5p suppresses tumorigenesis and metastasis of osteosarcoma through the p38 mitogen-activated protein kinases pathway by targeting transforming growth factor-beta 1

**DOI:** 10.1080/21655979.2022.2072619

**Published:** 2022-05-20

**Authors:** Haofeng Liang, Lin Li, Shuang Zhu, Jianye Tan, Bingsheng Yang, Xiaoping Wang, Guofeng Wu, Chao Xie, Lutao Li, Zhengwei Liu, Yucong Li, Haoqiang Song, Guoli Chen, Lijun Lin

**Affiliations:** a Department of Joint and Orthopedics, Zhujiang Hospital, Southern Medical University, Guangzhou, Guangdong Province, China; b Department of orthopedics, Huizhou Municipal Central Hospital, Huizhou, Guangdong Province, China; c Department of Orthopedics, Affiliated Hospital of Putian University, Putian, Fujian Province, China

**Keywords:** Osteosarcoma, miR-744-5p, TGFB1, p38 MAPK signaling pathway

## Abstract

Osteosarcoma (OS) is the most common malignant bone tumor in children and adolescents. Accumulating evidence has revealed that microRNAs (miRNAs) play a crucial role in the progression of OS. In this study, we found that miR-744-5p was the least expressed miRNA in patients with OS by analyzing GSE65071 from the GENE EXPRESSION OMNIBUS (GEO) database. Through real-time quantitative PCR (qRT-PCR), western blotting, colony formation assay, 5-Ethynyl-2-Deoxyuridine (EdU) incorporation assay, transwell migration, and invasion assays, we demonstrated its ability to inhibit the proliferation, migration, and invasion of OS cells in *vitro*. According to the luciferase reporter assay, transforming growth factor-β1 (TGFB1) was negatively regulated by miR-744-5p and reversed the effects of miR-744-5p on OS. Subcutaneous tumor-forming animal models and tail vein injection lung metastatic models were used in animal experiments, and it was found that miR-744-5p negatively regulated tumor growth and metastasis in *vivo*. Furthermore, rescue assays verified that miR-744-5p regulates TGFB1 expression in OS. Further experiments revealed that the p38 MAPK signaling pathway is involved in the miR-744-5p/TGFB1 axis. Generally, this study suggests that miR-744-5p is a negative regulator of TGFB1 and suppresses OS progression and metastasis via the p38 MAPK signaling pathway.

## Highlights

- miR-744-5p is lower expressed in osteosarcoma cells and tissue.
- miR-744-5p suppresses osteosarcoma development by targeting TGFB1.
- The p38 MAPK pathway is involved in the miR-744-5p/TGFB1 axis in osteosarcoma.

## 1. Introduction

Osteosarcoma (OS) is the most common malignant bone tumor in children and adolescents and originates from mesenchymal cells [1,2]. With a poor prognosis, the mortality rate could exceed 90% before polychemotherapy was introduced in clinical practice [3]. Significant progress has been made in the treatment of OS in the past 30 years, and effective therapies such as neoadjuvant chemotherapy combined with surgical resection have been introduced into clinical treatment. The prognosis and quality of life have visibly improved over the decades [4–6]. Nevertheless, the 5-year survival rate of patients with OS is still less than 50% [7]. Lung metastasis is the main problem for OS therapy, and the 5-year survival rate is <30% for metastatic OS [8]. Therefore, more potent therapeutic strategies and approaches for OS are urgently required.

The article "MicroRNA-744-5p suppresses tumorigenesis and metastasis of osteosarcoma through the p38 mitogen-activated protein kinases pathway by targeting transforming growth factor-beta 1" was retracted in 2026. Reasons: concerns about the data; concerns about the results or conclusions.

Epithelial-to-mesenchymal transition (EMT) is a complex process through which epithelial cells obtain the features of mesenchymal cells and lose their original polarity. This reversible phenotypic change is thought to stimulate tumor migration and invasion [9]. Accumulating evidence has revealed that EMT is closely related to tumor occurrence and development [10,11]. Therefore, suppressing EMT progression may be a potentially crucial approach for OS treatment.

MicroRNAs (miRNAs) are a family of endogenous small non-coding RNAs that regulate the expression of target genes by combining with 3 -untranslated regions (3’-UTRs) [12]. Accumulating evidence suggests that miRNAs play a crucial role in the occurrence and development of various tumors by regulating multiple signaling pathways [13,14]. Moreover, some miRNAs participate in the EMT process and regulate tumors [15,16]. miR-744-5p is upregulated in several tumors and is closely related to clinical characteristics [17–20]. However, the function of miR-744-5p in OS has not been reported, and the mechanism of action of miR-744-5p requires further study.

The MAPK pathway plays a crucial role in regulating partial miRNAs in various tumors [21–23]. As a member of the MAPK family, p38 MAPK participates in regulating proliferation, differentiation, and migration of various cells [24]. Previous studies have revealed that p38 could block the G2/M conversion through activating reactive oxygen species (ROS) [25]. Accumulating evidence have demonstrated that p38 MAPK pathway is involved in the progression of cancer, especially in the drug resistance [26–28]. Therefore, getting insight to the p38 MAPK is beneficial to oncotherapy.

Transforming growth factor-β (TGF-β), a prototype of the TGF-β family, with bifunctional regulation of cell proliferation, has been reported to have a promoting regulatory effect on EMT, and sufficient evidence has demonstrated that there is a conspicuous increase in the level of TGF-β in tumor cells [29,30]. Numerous studies have shown the correlation between TGFB1 and p38, moreover, TGFB1 could regulate the apoptosis together with the p38 MAPK pathway [31–33]. Nevertheless, the specific effects of TGFB1 on OS have not been clearly elucidated, and the detailed function of the TGFB1/p38 MAPK axis remains unclear.

The article "MicroRNA-744-5p suppresses tumorigenesis and metastasis of osteosarcoma through the p38 mitogen-activated protein kinases pathway by targeting transforming growth factor-beta 1" was retracted in 2026. Reasons: concerns about the data; concerns about the results or conclusions.

Based on this background, we hypothesized that miR-744-5p regulates the progression of OS. This study aimed to investigate the biofunction of miR-744-5p and determine its potential mechanisms. Through experiments in *vitro* and *vivo*, we found that miR-744-5p was remarkably downregulated in osteosarcoma, and it suppressed the proliferation, migration, and invasion of osteosarcoma cells by negatively regulating the TGFB1 and p38 MAPK signaling pathways. These findings may provide a new therapeutic strategy for osteosarcoma.

## 2. Materials and methods

### 2.1. Tissue samples

This study was approved by the Ethics Committee of the Second Affiliated Hospital of Southern Medical University. All human osteosarcoma and para-carcinoma samples were obtained from 25 patients who underwent biopsies before receiving chemotherapy and radiotherapy at the Department of Joint and Orthopedics. Tissue samples obtained from the biopsies were collected and immediately frozen in liquid nitrogen. The pathological and personal clinical information are listed in Table 1.

**Table 1.** Expression of miR-744-5p and TGFB1 according to patients’ clinical characteristics

		miR-744-5p expression			TGFB1 expression		
characteristics	total	Tumor tissue	para-carcinoma tissue	P value	Tumor tissue	para-carcinoma tissue	P value
Age (y)				0.291			0.377
< 18	14	0.93 ± 0.38	1.34 ± 0.40	0.024*	2.15 ± 0.86	1.24 ± 0.61	0.001***
≥ 18	11	0.91 ± 0.26	1.46 ± 0.47	0.017*	2.42 ± 0.65	1.42 ± 0.74	0.003**
Gender				0.391			0.374
Female	13	0.98 ± 0.37	1.30 ± 0.41	0.103	2.14 ± 0.77	1.40 ± 0.68	0.002**
Male	12	0.86 ± 0.27	1.56 ± 0.41	0.002**	2.41 ± 0.79	1.23 ± 0.66	0.001***
Location				0.572			0.531
Arm/hand	11	0.96 ± 0.32	1.72 ± 1.05	0.029*	2.38 ± 0.77	1.35 ± 0.66	0.004**
Leg/foot	14	0.89 ± 0.34	1.41 ± 0.44	0.015*	2.18 ± 0.80	1.30 ± 0.69	0.001***
TNM stage				0.135			0.014*
I	6	1.04 ± 0.25	1.26 ± 0.38	0.401	1.80 ± 0.60	1.21 ± 0.50	0.054
II	11	1.03 ± 0.30	1.40 ± 0.41	0.075	2.09 ± 0.67	1.27 ± 0.74	0.004**
III/IV	8	0.67 ± 0.29	1.59 ± 0.47	0.005**	2.88 ± 0.71	1.46 ± 0.72	0.003**
Tumor size				0.017*			0.014*
< 5 cm	11	1.09 ± 0.29	1.31 ± 0.41	0.272	1.86 ± 0.46	1.25 ± 0.53	0.001***
≥ 5 cm	14	0.89 ± 0.24	1.43 ± 0.43	0.006*	2.44 ± 0.84	1.37 ± 0.84	0.004**
Lung metastasis				0.005**			0.005**
Yes	8	0.67 ± 0.29	1.59 ± 0.47	0.005**	2.88 ± 0.71	1.46 ± 0.72	0.003**
No	17	1.04 ± 0.27	1.35 ± 0.39	0.043*	1.99 ± 0.64	1.25 ± 0.65	0.000***

### 2.2. Obtainment and analysis of original data

GES65071 from the GEO database was downloaded [34]. The R package affy was used for background correction and normalization. The R package limma was used to detect differences in miRNA expression levels between normal and OS samples. The filter criterion was log [fold change (FC)] > 1 and adjusted P-value  < 0.05 [35].

The article "MicroRNA-744-5p suppresses tumorigenesis and metastasis of osteosarcoma through the p38 mitogen-activated protein kinases pathway by targeting transforming growth factor-beta 1" was retracted in 2026. Reasons: concerns about the data; concerns about the results or conclusions.

### 2.3. Cells and cell culture

All human OS cells, including Saos-2, U-2 OS, MG-63, MNNG, 143 B, and the normal osteoblast cell line hFOB 1.19, were obtained from the American Type Culture Collection (ATCC, Manassas, US). OS cells were cultured in Dulbecco’s modified Eagle’s medium (DMEM; Invitrogen, US) supplemented with 10% fetal bovine serum (FBS) (Gibco, NY) and 1% penicillin/streptomycin (PS; Gibco, CA). The hFOB 1.19 cells were cultured in Dulbecco’s modified Eagle’s medium/Nutrient Mixture F-12 (DMEM/F12) (Life Technologies, NY) with 0.3 mgl/mL of G418, 10% FBS and 1% PS. All cells were incubated with 5% CO_2_ at 37°C.

### 2.4. Establishment of transfected cells

Plasmids overexpressing miR-744-5p and TGFB1 were used in in vitro experiments. The cells were cultured in 6-well plates. After washing with DMEM, the complex liquid was added to the plates and incubated for 24 h. The cells were then cultured in DMEM containing 10% FBS for 48 h. G418 selective media was used to screen out the transfected cells. The lentiviral transfection was performed in vivo. The cells were cultured in 24-well plates for 24 h. Medium with 2 μg/ml polybrene was used to replace the original medium, and lentivirus transfected with miR-744-5p or TGFB1 was added into the wells. After incubation for 24 h, cells were cultured in DMEM for another 72 h. Transfection efficiency was examined using qRT-PCR.

### 2.5. Quantitative real-time PCR (qRT-PCR)

According to the manufacturer’s protocol, total RNAs from cells and tissue samples in Trizol (Invitrogen, US) were extracted from the frozen pulverized samples. Total RNA (500 ng) was reverse-transcribed into cDNA. The cDNA was diluted five times with enzyme-free water. One-step qRT-PCR was performed in a 10 µL reaction system. The purity and integrity of the total RNAs were examined through absorption at 260 nm and 280 nm. Primers for TGFB1, U6, and GAPDH were purchased from TsingKe (Beijing, China), and the primers for miR-744-5p were designed based on the purchased primers. Reverse transcription was performed using the SuperScriptTM Preamplification System for First Strand cDNA Synthesis according to the manufacturer’s protocol, and qPCR was performed using a LightCycler® Real-Time PCR; U6 and GAPDH served as endogenous controls. The sequences of the primers were as follows: TGFB1 forward, 5′-GGCCAGATCCTGTCCAAGC-3′; TGFB1 reverse, 5′-GTGGGTTTCCACCATTAGCAC-3′; GADPH forward, 5′-GGAGCGAGATCCCTCCAAAAT-3′; GAPDH reverse, 5′-GGCTGTTGTCATACTTCTCATGG-3′; U6 forward, 5′-CTCGCTTCGGCAGCACA-3′; U6 reverse, 5′-AACGCTTCACGAATTTGCGT-3′; miR-744-5p forward, 5′-AATGCGGGGCTAGGGCTA-3′; miR-744-5p reverse, 5′-GTGCAGGGTCCGAGGT-3′.

The article "MicroRNA-744-5p suppresses tumorigenesis and metastasis of osteosarcoma through the p38 mitogen-activated protein kinases pathway by targeting transforming growth factor-beta 1" was retracted in 2026. Reasons: concerns about the data; concerns about the results or conclusions.

### 2.6. Western blotting (WB)

Proteins were extracted from the cells, and the protein concentration was assessed using the BCA protein assay kit (Beyotime, China). The proteins were electrophoresed through 10% SDS-PAGE for 4 h at 40 volts and then transferred to PVDF membranes. Proteins were incubated with specific primary antibodies at 4°C overnight. After washing with TBST, the proteins were incubated with secondary antibodies at room temperature for 2 h. Rat anti-TGFB1 (1:1000, Abcam), GAPDH (1: 10,000, Proteintech), N-cadherin (1:1000, Abcam), E-cadherin (1:1000, Abcam), vimentin (1:1000, Abcam), p-P38 (1:1000, Abcam), and t-P38 (1:1000, Abcam) antibodies were used to detect the proteins. Reacting bands were acquired with ECL reagent, and quantitative analysis was performed with ImageJ normalized to GAPDH.

### 2.7. Colony formation assay

Approximately 800 OS cells were seeded into a six-well plate and cultured with DMEM and 10% FBS at 37°C for 1 week. When colonies became invisible, they were washed with PBS, fixed with 4% paraformaldehyde, and stained with 0.1% crystal violet. Images were captured using a scanner, and counts were calculated manually.

5-Ethynyl-2-Deoxyuridine (EdU) incorporation assay

The EdU incorporation assays were performed according to the manufacturer’s protocol. OS cells (1 × 104 cells/well of OS cells were seeded in 96-well plates and cultured in 100 μl of 50 μM EdU medium for 2 h. The cells were then fixed with 4% paraformaldehyde and destained with 2 mg/mL glycine. Next, Apollo staining was performed with 1X Apollo dyeing reaction fluid. A 1X Hoechst 33,342 reaction mixture was used for DNA staining. At least 50 cells per well were randomly selected. The intensity was measured in five random fields, and photos were taken with a fluorescence microscope (Carl Zeiss, Germany).

### 2.8. Transwell migration and invasion assay

Transwell migration assay was performed to detect cell migratory ability. A total of 4.0 × 104 cells were seeded in the upper chamber with 200 µL of DMEM, whereas the lower chamber was immersed in 600 µL of DMEM with 10% FBS. After incubation for 24 h, the lower chamber was removed, and the cells were fixed with 4% paraformaldehyde for 30 min. The cells were then stained with 0.1% crystal violet for 20 min, and the non-migratory cells in the upper chamber were wiped with a swab. After removing crystal violet, five randomized fields were observed and photographed under a microscope. For the transwell invasion assay, Matrigel (BD 5 mg/ml) was diluted to 1 mg/ml in a serum-free medium. The resulting matrigel (100 μl of resulting Matrigel was placed in the upper chamber and incubated at 37°C for 1 h. The following steps were the same as those used in the transwell migration assay.

The article "MicroRNA-744-5p suppresses tumorigenesis and metastasis of osteosarcoma through the p38 mitogen-activated protein kinases pathway by targeting transforming growth factor-beta 1" was retracted in 2026. Reasons: concerns about the data; concerns about the results or conclusions.

### 2.9. Luciferase reporter assay

Possible miR-744-5p-binding sites were obtained from the miRDB database. Wild-type TGFB1 (WT-TGFB1-3’-UTR) and mutant TGFB1 (MUT-TGFB1-3’-UTR) were synthesized by GenePharma (Shanghai, China). Cells overexpressing miR-744-5p were transfected with the WT-TGFB1-3’-UTR, and the negative controls were transfected with the MUT-TGFB1-3’-UTR. 48 h later, after transfection, luciferase activity was determined using the Dual-Luciferase Assay System (Promega, Madison, WI, US) and normalized to Renilla luciferase.

### 2.10. Immunohistochemistry (IHC)

The slides were immersed in miscible liquids of potassium dichromate and concentrated sulfuric acid and then flushed for 1 h. Polylysine was smeared on the surface. The tissues were then embedded in paraffin. The tissue sections were deparaffinized with xylene and ethanol. The sections were immersed in 0.01 mol/L sodium citrate buffer for 10 min and 3% hydrogen peroxide for 30 min at room temperature. The sections were then placed in phosphate-buffered saline (PBS) for 5 min and sealed with 5% bovine serum for 0.5 h at 37°C. The tissue sections were incubated with primary antibodies overnight at 4°C. After washing three times with PBS, the sections were incubated with secondary antibodies for 0.5 h at 37°C and then incubated with SABC for another 0.5 Â h. After wiping up the sections, color developing agents were added, followed by hematoxylin staining. Finally, the sections were dehydrated with ethanol and xylene and sealed with resinence. The primary antibodies used were Ki-67, E-cadherin, N-cadherin, and vimentin (Abcam, Cambridge, UK). Images were captured using an orthophoto microscope.

### 2.11. Hematoxylin-eosin (HE) staining

Tissues were immersed in a stationary liquid containing 10% methanol. After dehydration with ethanol and xylene, samples were embedded in paraffin. The sections were deparaffinized with xylene and ethanol before staining. The sections were successively immersed in hematoxylin, hydrochloric acid, and ammonium hydroxide and flushed with distilled water for 1 h. Next, the sections were dehydrated in ethanol and dipped in an eosin staining solution. Finally, the sections were immersed in ethanol and xylene and sealed with gum.

### 2.12. Animal experiments

Nude mice were purchased from the Animal Core Facility of Southern Medical University and were randomly divided into five groups, 5 in each group. OS cells with RFP were inoculated into the subcutaneous tissue of nude mice. Pulmonary metastasis models were developed by tail vein injection. The volume and size of the tumors were recorded every three days, and the tumors were separated and imaged on day 28th. Mice were sacrificed at the end of the experiment.

The article "MicroRNA-744-5p suppresses tumorigenesis and metastasis of osteosarcoma through the p38 mitogen-activated protein kinases pathway by targeting transforming growth factor-beta 1" was retracted in 2026. Reasons: concerns about the data; concerns about the results or conclusions.

### 2.13 Statistical analysis

All experiments were repeated at least three times, and data were presented as mean ± standard deviation. Independent Student’s t-test and one-way analysis ANOVA were used to compare the differences in clinical characteristics between the two groups. A paired t-test was used to evaluate differences in miRNA expression between TGFB1 and miR-744-5p in tissue samples. Pearson’s chi-square test was used to detect the relationship between miR-744-5p and TGFB1. A log-rank test was conducted to evaluate the prognosis and OS of patients with OS. Statistical analyses were performed using SPSS, v. 23.0. Statistical significance was set at p < 0.05. Data were presented as mean ± SD. * p < 0.05, ** p < 0.01, *** p < 0.001 [36].

## 3. Results

In this study, we investigated the correlation between miR-744-5p and OS and how miR-744-5p regulated TGFB1 and p38 MAPK pathways. Bioinformatics analysis was performed to detect differentially expressed miRNAs and the potential mechanisms involved in OS. Using colony formation, EdU, transwell migration, and invasion assays, we evaluated whether miR-744-5p affected OS cell proliferation, migration, and invasion in *vitro*. A subcutaneous tumor model of nude mice was used in the animal experiments. The size and volume of the tumor, immunohistochemical staining, and hematoxylin and eosin staining were used to investigate the function of miR-744-5p in *vivo*. Rescue assays were performed to determine the correlation between TGFB1 and miR-744-5p in *vitro* and *vivo*.

### 3.1. miR-744-5p was downregulated in OS cells and tissues

To investigate the expression of miRNAs in OS cells and tissue samples, GSE65071 from the GEO database was analyzed using the R package. A volcano plot demonstrated differences in miRNA expression between OS and normal tissues (Figure 1a). According to the miRNA expression levels, the up-and downregulated miRNAs are displayed on a cluster heat map (Figure 1b). Eighty-nine miRNAs were downregulated in OS tissues compared to normal tissues (fold change > 1, FDR < 0.05), and the top 10 downregulated miRNAs are shown in Figure 1c. We found that miR-744-5p was the most downregulated miRNA among these miRNAs. Based on these results, we attempted to determine the specific function of miR-744-5p in OS. Low expression of miR-744-5p was found in OS cells, including 143 B, MNNG, U-2 OS, MG-63, and Saos-2, compared with the hFOB 1.19 cell line (Figure 1d). Furthermore, qRT-PCR was performed to assess miR-744-5p expression in 25 paired OS and adjacent normal tissues, and the results showed that miR-744-5p was significantly downregulated in the OS tissues (Figure 1e).

The article "MicroRNA-744-5p suppresses tumorigenesis and metastasis of osteosarcoma through the p38 mitogen-activated protein kinases pathway by targeting transforming growth factor-beta 1" was retracted in 2026. Reasons: concerns about the data; concerns about the results or conclusions.

**Figure 1.** miR-744-5p is downregulated in osteosarcoma cell lines and clinical tissues. (a) Volcano plot demonstrated the expressive diversity of miRNAs between OS and normal tissues from GSE65071. (b) The cluster heat map showed the upregulated and downregulated miRNAs in GSE65071. (c) The top 10 downregulated miRNAs are listed. (d) The relative expression of miR-744-5p was remarkably suppressed in OS cell lines. (e) Expression of miR-744-5p was significantly downregulated in OS clinical tissues than in para-carcinoma tissues. * p < 0.05, ** p < 0.01, *** p < 0.001.

### 3.2. miR-744-5p was closely related to better clinical characteristics of patients with OS

As shown in (Figure 2a-d), the expression level was significantly associated with OS clinical characteristics; higher expression of miR-744-5p was found in patients with earlier pathological stages, smaller tumor size, localized growth, and higher long-term survival rate. Detailed clinical data are shown in Table 1.

**Figure 2.** miR-744-5p is closely related to the clinical features of patients with OS. (a) Lower expression of miR-744-5p was found in the middle and advanced stage of OS compared to the early stage. (b) Lower expression of miR-744-5p was related to larger tumors. (c) Lower expression of miR-744-5p was found in more patients with metastasis. (d) Log-Rank test demonstrated that patients with higher miR-744-5p expression had a better prognosis. * p < 0.05, ** p < 0.01, *** p < 0.001.

### 3.3. *Upregulation of miR-744-5p inhibited OS cell proliferation, invasion and migration* in vitro

MG-63 and 143 B cells were used for further in vitro experiments. qRT-PCR was performed to evaluate the transfection efficiency of miR-744-5p mimics (Figure 3a). Colony formation and EdU assays were performed to detect the effect of miR-744-5p on cell proliferation. Figure 3b-e demonstrated that overexpressed miR-744-5p significantly inhibited OS cell proliferation. Transwell migration assays were performed to assess the influence of miR-744-5p on the migratory ability of OS cells in vitro, and the results showed that the overexpression of miR-744-5p significantly decreased the migration of OS cells. Similarly, the invasive ability of OS cells was detected by Transwell invasion assays, and upregulation of miR-744-5p suppressed the invasive ability of both 143 B and MG-63 cells (figure 3f-i). Furthermore, WB analysis demonstrated that miR-744-5p decreased the expression of the proteins, N-cadherin and vimentin, and increased the level of E-cadherin in both MG-63 and 143 B OS cells (Figure 3j-l).

The article "MicroRNA-744-5p suppresses tumorigenesis and metastasis of osteosarcoma through the p38 mitogen-activated protein kinases pathway by targeting transforming growth factor-beta 1" was retracted in 2026. Reasons: concerns about the data; concerns about the results or conclusions.

**Figure 3.** Overexpression of miR-744-5p suppressed OS cells EMT, migration and invasion in vitro. (a) miR-744-5p mimics were successfully transfected into 143B and MG-63 cell lines. (b-e) Colony formation and EdU assays demonstrated that overexpression of miR-744-5p suppressed the proliferation of OS cells. (f-i) Transwell migration and invasion assays showed that overexpressed miR-744-5p remarkably inhibited the migratory and invasive ability of OS cells. (j-l) WB indicated that overexpression of miR-744-5p suppressed the expression level of metastasis-related proteins in OS cells. * p < 0.05, ** p < 0.01, *** p < 0.001.

### 3.4. *miR-744-5p suppressed xenograft tumor growth and metastasis* in vivo

To investigate the effect of miR-744-5p in vivo, OS cells transfected with Lv-miR-NC or Lv-miR-744-5p were implanted subcutaneously in nude mice. Figure 4a shows the metastatic tumor obtained from mice sacrificed at week 4. The tumor volume was smaller and the average weight lower in the Lv-miR-744-5p group than in the NC group (Figure 4b, c). IHC was performed to assess the expression of proliferation- and invasion-related factors, including Ki-67, E-cadherin, N-cadherin, and vimentin. The results demonstrated that Ki-67, N-cadherin, and vimentin were downregulated in the Lv-miR-744-5p group compared to the controls, indicating that miR-744-5p suppressed OS cell proliferation and invasion of OS cells in vivo. In contrast, E-cadherin expression was higher in the Lv-miR-NC group than in the Lv-miR-NC group (Figure 4d, e). Less OS cells were observed in the miR-744-5p overexpressing group as determined by HE staining (figure 4f, g).

**Figure 4.** miR-744-5p suppressed xenograft tumor growth and pulmonary metastasis in vivo. (a-c) miR-744-5p mimics suppressed the tumor growth in nude mice, and the volume and weight were smaller and lighter compared to the miR-744-5p-NC group. (d, e) Higher expression of E-cadherin and lower expression of Ki-67, N-cadherin and vimentin were found in the Lv-miR-744-5p group according to IHC. (f, g) The HE staining demonstrated that less OS cells were found in the lungs of nude mice of the Lv-miR-744-5p group, indicating that miR-744-5p suppressed pulmonary metastasis. * p < 0.05, ** p < 0.01, *** p < 0.001.

### 3.5. TGFB1 was upregulated in OS tissues and was a target of miR-744-5p

The main function of miRNAs is to inhibit translation or promote the degradation of target genes. Thus, we attempted to determine the downstream mechanism of miR-744-5p in the occurrence and development of OS. The miRDB database was checked, and 111 genes were found to be potential targets of miR-744-5p. KEGG pathway enrichment analysis demonstrated that the MAPK signaling pathway was the center of most of the mentioned genes(Figure 5a). Among all candidate genes in the MAPK axis, TGFB1 was downregulated by miR-744-5p overexpression in both 143 B and MG-63 OS cells (Figure 5b, c). A luciferase reporter assay was performed to detect the specific relationship between TGFB1 and miR-744-5p. Results showed that miR-744-5p directly targeted TGFB1 and overexpressed miR-744-5p significantly suppressed the luciferase activity of OS cells (Figure 5d, e). WB verified that miR-744-5p negatively regulated the expression of TGFB1, and MAPK-related proteins were downregulated in the miR-744-5p mimic group (figure 5f-h). qRT-PCR was performed to investigate the expression of TGFB1 in OS cell lines and tissue samples. Higher expression of TGFB1 was found in various OS cells, especially in MG-63 and 143 B cells, and TGFB1 expression was significantly higher in OS tissues than in adjacent tissues (Figure 5i, j). Furthermore, TGFB1 was negatively correlated with miR-744-5p, with an r of −0.7326 in OS tissues (Figure 5k).

The article "MicroRNA-744-5p suppresses tumorigenesis and metastasis of osteosarcoma through the p38 mitogen-activated protein kinases pathway by targeting transforming growth factor-beta 1" was retracted in 2026. Reasons: concerns about the data; concerns about the results or conclusions.

**Figure 5.** TGFB1 expression was upregulated in OS cell lines and tissues and was a target of miR-744-5p. (a) miRDB database demonstrated 111 genes targeted to miR-744-5p, and the MAPK signaling pathway was the most relative one according to the KEGG pathway enrich the analysis. (b, c) Among all candidate genes in the MAPK axis, TGFB1 was significantly downregulated by miR-744-5p both in 143B and MG-63 cells at the same time. (d, e) The WT-TGFB1-3’-UTR and MUT-TGFB1-3’-UTR were synthesized. Overexpressed miR-744-5p significantly suppressed the luciferase activity of WT-TGFB1-3’-UTR but had no effect on MUT-TGFB1-3’-UTR in 143B and MG-63 cells. (f-h) WB showed that miR-744-5p downregulated the expression level of TGFB1 and p-P38. (i) Higher expression of TGFB1 was found in OS cell lines, especially in 143B and MG-63 cells. (j) Expression of TGFB1 was significantly upregulated in OS clinical tissues than para-carcinoma tissues. (k) TGFB1 expression level was negatively related to miR-744-5p in OS tissues. * p < 0.05, ** p < 0.01, *** p < 0.001.

### 3.6. TGFB1 was connected with poor clinical characteristics of OS patients

qRT-PCR was conducted to determine the relationship between TGFB1 expression and clinical characteristics. Figure 6a-c demonstrated that higher expression levels of TGFB1 were found in more patients with advanced, larger, and metastatic tumors. Although there was no statistical difference in overall survival, patients with a higher expression level of TGFB1 tend to have a poorer prognosis (Figure 6d).

The article "MicroRNA-744-5p suppresses tumorigenesis and metastasis of osteosarcoma through the p38 mitogen-activated protein kinases pathway by targeting transforming growth factor-beta 1" was retracted in 2026. Reasons: concerns about the data; concerns about the results or conclusions.

**Figure 6.** TGFB1 is related to the clinical features of patients with OS. (a) Higher expression of TGFB1 was found in the middle and advanced stage of OS compared to the early stage. (b) Higher expression of TGFB1 was related to larger tumors. (c) Higher expression of TGFB1 was found in more patients with metastasis. (d) Although there was no statistical difference in overall survival between the two groups, patients with a lower expression level of TGFB1 tend to have a better prognosis. * p < 0.05, ** p < 0.01, *** p < 0.001.

### 3.7. *miR-744-5p suppressed OS proliferation, migration and invasion by regulating MAPK signaling pathway through TGFB1* in vitro

To verify that miR-744-5p regulates proliferation, migration, and invasion of OS cells through TGFB1, a series of rescue experiments showed that TGFB1 was overexpressed artificially, and qRT-PCR showed TGFB1 was successfully transfected into OS cells (Figure 7a). Colony formation and EdU assays revealed that overexpression of miR-744-5p significantly suppressed the proliferation of OS cells, and the effects were restored by the upregulation of TGFB1 (Figure 7b-f). Transwell migration and invasion assays were performed, and results revealed that TGFB1 reversed the protective effects of miR-744-5p on OS migration and invasion (Figure 7g-j). WB was performed to detect the downstream mechanism of the miR-744-5p/TGFB1 axis in OS cells. Figure 7k-n showed that overexpressed miR-744-5p inhibited the expression of N-cadherin, vimentin, TGFB1, and t-P38, and promoted the expression of E-cadherin, indicating that EMT and MAPK pathways play essential roles in the regulation of OS by the miR-744-5p/TGFB1 axis.

**Figure 7.** miR-744-5p downregulated MAPK signaling pathway through inhibiting TGFB1 expression. (a) TGFB1 was successfully transfected into 143B and MG-63 cell lines. (b-f) Colony formation and EdU assays demonstrated that miR-744-5p suppressed the proliferation of OS cells, and overexpression of TGFB1 could reverse the effect. (g-j) Transwell migration and invasion assays indicated that overexpressed miR-744-5p significantly suppressed the migratory and invasive ability of OS cells, and overexpressed TGFB1 could abolish the influence. (k-n) Western blotting assays showed that miR-744-5p downregulated metastasis-related, MAPK-related and TGFB1 proteins in OS cells, while TGFB1 own contrary functions. * p < 0.05, ** p < 0.01, *** p < 0.001.

The article "MicroRNA-744-5p suppresses tumorigenesis and metastasis of osteosarcoma through the p38 mitogen-activated protein kinases pathway by targeting transforming growth factor-beta 1" was retracted in 2026. Reasons: concerns about the data; concerns about the results or conclusions.

### 3.8. *miR-744-5p suppressed OS growth and metastasis by regulating MAPK signaling pathway through TGFB1* in vivo

Rescue assays were performed to verify the role of miR-744-5p and TGFB1 in vivo. OS cells transfected with Lv-miR-NC, Lv-miR-744-5p, or Lv-miR-744-5p with TGFB1 were implanted subcutaneously into nude mice. Figure 8a-c demonstrates that overexpression of miR-744-5p suppressed the growth of tumors, and there was a significant difference in weight and volume; however, the introduction of TGFB1 inhibited the effects of miR-744-5p, making tumors remarkably larger and heavier. Moreover, IHC showed that higher TGFB1 expression increased the expression level of ki-67, N-cadherin, and vimentin, which were downregulated by miR-744-5p (Figure 8d, e). figure 8f, g demonstrates that Lv-miR-744-5p inhibited the invasion of OS cells, while the inverse overexpression of TGFB1 promoted metastasis conspicuously.

**Figure 8.** miR-744-5p suppressed tumor growth and pulmonary metastasis through TGFB1 in vivo. (a-c) miR-744-5p inhibited metastasis and growth of xenograft tumors, and TGFB1 reversed the effects of miR-744-5p. (d, e) IHC showed that TGFB1 upregulated the expression level of Ki-67, N-cadherin and vimentin, which were suppressed in the miR-744-5p mimics group. (f, g) TGFB1 promoted the decreased pulmonary metastasis caused by miR-744-5p. * p < 0.05, ** p < 0.01, *** p < 0.001.

## 4. Discussion

OS is the most frequent primary malignant tumor of the bones, which occurs in adolescents [37]. However, although accumulating research has been conducted, OS’ poor prognosis has not been well established. Therefore, it is necessary to develop novel therapeutic targets for OS treatment.

miRNAs have been reported to be directly related to the regulation of gene expression, and substantial evidence has revealed that abnormal miRNA expression occurs in numerous tumors [38–40]. Numerous studies have shown that various miRNAs have different functions in developing OS [41–44]. Shen L et al. [45] demonstrated that miR-217 suppresses OS progression and metastasis through regulating the expression of WASF3. In contrast, miR-652 promotes tumorigenesis and metastasis by targeting RORA [46]. miR-744-5p has been reported to play a negative regulatory role in some cancers, such as ovarian cancer and non-small cell lung cancer; however, few studies have investigated the effects and mechanism of miR-744-5p in OS [17–19]. In accordance with the data from the GEO database and qRT-PCR results, we found that miR-744-5p was downregulated in OS cells and tissue samples, which is consistent with previous studies.

EMT participates in the migration and invasion of tumor cells and promotes cancer progression and metastasis. During EMT, epithelial cancer cells acquire the characteristics of mesenchymal cells and lose polarity and adhesion between cells. These features accelerate the migration and invasion of OS cells, promote tumor metastasis, and increase drug resistance in OS therapies [47–49]. Furthermore, reduction in E-cadherin and induction of N-cadherin and vimentin levels have been reported in converting epithelial cells to mesenchymal cells [50,51]. In this study, a series of experiments were performed to investigate the function and molecular mechanism of miR-744-5p in OS. We found that miR-744-5p was expressed at low levels in OS tissues and played a negative regulatory role in tumor development. Results indicated that miR-744-5p downregulated the cell proliferation, migration and invasion of OS and could be a novel target in the treatment of OS. Moreover, via luciferase reporter assay, we proved that there was a binding sequence between miR-744-5p and TGFB1, and TGFB1 was found to be suppressed by miR-744-5p in the study.

The article "MicroRNA-744-5p suppresses tumorigenesis and metastasis of osteosarcoma through the p38 mitogen-activated protein kinases pathway by targeting transforming growth factor-beta 1" was retracted in 2026. Reasons: concerns about the data; concerns about the results or conclusions.

TGFB1, a regulatory cytokine that participates in multiple signaling pathways, has been reported to play dual roles in cell growth by regulating cell autophagy [52]. TGFB1 acts as a tumor suppressor in the early stage of tumors or normal tissues and promotes tumorigenesis and metastasis in advanced tumors [29,53,54]. Recent studies have demonstrated that TGFB1 plays a vital role in the progression of various tumors, including ovarian, colorectal, cervical, and gastric cancers [29,53,55–57]. It was also found that TGFB1 induces EMT during tumorigenesis and metastasis in cancer [58,59]. In this study, we found that TGFB1 was significantly upregulated in tumor tissues and highly correlated with OS development, indicating that TGFB1 could play a stimulatory role in tumorigenesis and metastasis in OS. Moreover, the relationship between clinical characteristics and TGFB1 was verified in this study, and the results demonstrated that a high expression level could result in a poor prognosis for patients with OS, which was quite similar to other related studies [60,61].

Through bioinformatic analysis, we found that the MAPK signaling pathway was remarkably correlated with miR-744-5p. To determine the specific mechanism of this axis in OS, we performed various experiments. WB demonstrated that overexpression of miR-744-5p significantly suppressed EMT-related and p38 MAPK-related proteins in both 143 B and MG-63 OS cells. Moreover, TGFB1 was overexpressed in the miR-744-5p overexpressed group, and the results revealed a trend back to that of the control group. Similar results were observed in rescue assays in vivo. P38 belongs to the MAPK family, and the p38 MAPK signaling pathway is thought to be a central section that regulates apoptosis in cells [62]. The function of p38 MAPK pathway in OS still need further investigation, Zhang L et al. [63] revealed that activation of p38 pathway was conducive to inhibiting the progression of OS. While Shi D et al. [64] regarded p38 MAPK as a key part in promoting tumorigenesis in OS. In this study, we found that the phosphorylation of p38 was suppressed with the overexpression of miR-744-5p, and was positively correlated with TGFB1, indicating that p38 MAPK could facilitate the progression of OS in miR-744-5p/TGFB1 axis.

The article "MicroRNA-744-5p suppresses tumorigenesis and metastasis of osteosarcoma through the p38 mitogen-activated protein kinases pathway by targeting transforming growth factor-beta 1" was retracted in 2026. Reasons: concerns about the data; concerns about the results or conclusions.

This study had some limitations. We constructed OS mouse models through subcutaneous injection due to the limitation of experimental conditions, and orthotopic models were used to examine the results in further studies. Furthermore, a functional deficiency assay was performed to verify the effects of miR-744-5p and TGFB1. In recent years, liquid biopsy has been recognized as a convenient and efficacious checkup method, and miRNAs have been detected in multiple body liquids [65,66]. miRNAs could be a potential therapeutic target in the treatment of cancers, and expression profile analysis of miRNAs in body liquids could be conducted to determine whether miR-744-5p could be utilized in the clinical treatment of patients with OS.

This study is the first to reveal the relationship between miR-744-5p and OS. Patients with OS with a high expression level of miR-744-5p were found to have better clinical characteristics and prognosis, indicating that miR-744-5p could be a latent target in prediction and assessment during treatment. We detected the downstream mechanism of miR-744-5p and found that TGFB1 was a target gene of the miRNA and that the p38 MAPK signaling pathway was involved in this process.

## 5. Conclusions

In conclusion, we found that miR-744-5p was negatively related to the progression and metastasis of osteosarcoma via the downregulation of TGFB1 through the p38 MAPK signaling pathway. We demonstrated that miR-744-5p suppresses OS cells’ proliferation, migration, and invasion through the p38 MAPK signaling pathway by directly targeting TGFB1. Thus, the miR-744-5p/TGFB1 signaling pathway could be a potential therapeutic target for OS and may provide further insight into the molecular mechanism of OS.

## Data Availability

The datasets generated and analyzed during the current study are available in the [GEO DataSets] repository, [https://www.ncbi.nlm.nih.gov/geo/query/acc.cgi?acc=GSE65071].

## References

[1] Bishop MW, Janeway KA, Gorlick R. Future directions in the treatment of osteosarcoma. Curr Opin Pediatr. 2016;28(1):26–33.2662655810.1097/MOP.0000000000000298PMC4761449

The article "MicroRNA-744-5p suppresses tumorigenesis and metastasis of osteosarcoma through the p38 mitogen-activated protein kinases pathway by targeting transforming growth factor-beta 1" was retracted in 2026. Reasons: concerns about the data; concerns about the results or conclusions.

[2] Lindsey BA, Markel JE, Kleinerman ES. Osteosarcoma overview. Rheumatol Ther. 2017;4(1):25–43.2793346710.1007/s40744-016-0050-2PMC5443719

[3] Ritter J, Bielack SS. Osteosarcoma. Ann Oncol. 2010;21(7):vii320–325.2094363610.1093/annonc/mdq276

[4] Harrison DJ, Geller DS, Gill JD, et al. Current and future therapeutic approaches for osteosarcoma. Expert Rev Anticancer Ther. 2018;18(1):39–50.2921029410.1080/14737140.2018.1413939

[5] Reed DR, Hayashi M, Wagner L, *et al*. Treatment pathway of bone sarcoma in children, adolescents, and young adults. Cancer. 2017;123(12):2206–2218.2832333710.1002/cncr.30589PMC5485018

[6] Tsukamoto S, Errani C, Angelini A, et al. Current treatment considerations for osteosarcoma metastatic at presentation. Orthopedics. 2020;43(5):e345–e358.3274521810.3928/01477447-20200721-05

[7] Kager L, Tamamyan G, Bielack S. Novel insights and therapeutic interventions for pediatric osteosarcoma. Future Oncol. 2017;13(4):357–368.2765103610.2217/fon-2016-0261

[8] Mirabello L, Troisi RJ, Savage SA. International osteosarcoma incidence patterns in children and adolescents, middle ages and elderly persons. Int J Cancer. 2009;125(1):229–234.1933084010.1002/ijc.24320PMC3048853

[9] Zhang Y, Weinberg RA. Epithelial-to-mesenchymal transition in cancer: complexity and opportunities. Front Med. 2018;12(4):361–373.3004322110.1007/s11684-018-0656-6PMC6186394

[10] Chen T, You Y, Jiang H, et al. Epithelial-mesenchymal transition (EMT): a biological process in the development, stem cell differentiation, and tumorigenesis. J Cell Physiol. 2017;232(12):3261–3272.2807925310.1002/jcp.25797PMC5507753

[11] Suarez-Carmona M, Lesage J, Cataldo D, et al. EMT and inflammation: inseparable actors of cancer progression. Mol Oncol. 2017;11(7):805–823.2859910010.1002/1878-0261.12095PMC5496491

[12] Aigner A. MicroRNAs (miRNAs) in cancer invasion and metastasis: therapeutic approaches based on metastasis-related miRNAs. J Mol Med (Berl). 2011;89(5):445–457.2123453310.1007/s00109-010-0716-0

[13] Rupaimoole R, Slack FJ. MicroRNA therapeutics: towards a new era for the management of cancer and other diseases. Nat Rev Drug Discov. 2017;16(3):203–222.2820999110.1038/nrd.2016.246

[14] Wang C, Tang Z, Zhang Z, et al. MiR-7-5p suppresses invasion via downregulation of the autophagy-related gene ATG7 and increases chemoresistance to cisplatin in BCa. Bioengineered. 2022;13(3):7328–7339.3530057210.1080/21655979.2022.2037323PMC9278970

[15] Jaca A, Govender P, Locketz M, et al. The role of miRNA-21 and epithelial mesenchymal transition (EMT) process in colorectal cancer. J Clin Pathol. 2017;70(4):331–356.2767221710.1136/jclinpath-2016-204031

The article "MicroRNA-744-5p suppresses tumorigenesis and metastasis of osteosarcoma through the p38 mitogen-activated protein kinases pathway by targeting transforming growth factor-beta 1" was retracted in 2026. Reasons: concerns about the data; concerns about the results or conclusions.

[16] Suzuki HI. MicroRNA control of TGF-beta signaling. Int J Mol Sci. 2018;19(7):1901.10.3390/ijms19071901PMC607362629958433

[17] Chen S, Shi F, Zhang W, et al. miR-744-5p inhibits non-small cell lung cancer proliferation and invasion by directly targeting PAX2. Technol Cancer Res Treat. 2019;18:1533033819876913.3152260710.1177/1533033819876913PMC6747846

[18] Yuan Q, Fan Y, Liu Z, et al. miR-744-5p mediates lncRNA HOTTIP to regulate the proliferation and apoptosis of papillary thyroid carcinoma cells. Exp Cell Res. 2020;392(1):112024.3233502910.1016/j.yexcr.2020.112024

[19] Zhang W, Liao K, Liu D. MicroRNA7445p is downregulated in colorectal cancer and targets SEPT2 to suppress the malignant phenotype. Mol Med Rep. 2021;23(1):54.3320080210.3892/mmr.2020.11692PMC7705998

[20] Zhao LG, Wang J, Li J, et al. miR-744-5p inhibits cellular proliferation and invasion via targeting ARF1 in epithelial ovarian cancer. Kaohsiung J Med Sci. 2020;36(10):799–807.3255834510.1002/kjm2.12253PMC11896257

[21] Lee S, Rauch J, Kolch W. Targeting MAPK signaling in cancer: mechanisms of drug resistance and sensitivity. Int J Mol Sci. 2020;21(3):1102.10.3390/ijms21031102PMC703730832046099

[22] Miao LJ, Yan S, Zhuang QF, et al. miR-106b promotes proliferation and invasion by targeting Capicua through MAPK signaling in renal carcinoma cancer. Onco Targets Ther. 2019;12:3595–3607.3119086210.2147/OTT.S184674PMC6525582

[23] Wang L, Sun L, Wang Y, et al. miR-1204 promotes hepatocellular carcinoma progression through activating MAPK and c-Jun/AP1 signaling by targeting ZNF418. Int J Biol Sci. 2019;15(7):1514–1522.3133798010.7150/ijbs.33658PMC6643133

[24] Wagner EF, Nebreda AR. Signal integration by JNK and p38 MAPK pathways in cancer development. Nat Rev Cancer. 2009;9(8):537–549.1962906910.1038/nrc2694

[25] Liu W, Ning R, Chen RN, *et al*. Aspafilioside B induces G2/M cell cycle arrest and apoptosis by up-regulating H-Ras and N-Ras via ERK and p38 MAPK signaling pathways in human hepatoma HepG2 cells. Mol Carcinog. 2016;55(5):440–457.2568370310.1002/mc.22293

[26] Jie Z, Xie Z, Zhao X, et al. Glabridin inhibits osteosarcoma migration and invasion via blocking the p38- and JNK-mediated CREB-AP1 complexes formation. J Cell Physiol. 2019;234(4):4167–4178.3014672310.1002/jcp.27171

[27] Rasmussen MH, Lyskjaer I, Jersie-Christensen RR, et al. miR-625-3p regulates oxaliplatin resistance by targeting MAP2K6-p38 signalling in human colorectal adenocarcinoma cells. Nat Commun. 2016;7:12436.2752678510.1038/ncomms12436PMC4990699

[28] Wen S, Hou Y, Fu L, et al. Cancer-associated fibroblast (CAF)-derived IL32 promotes breast cancer cell invasion and metastasis via integrin beta3-p38 MAPK signalling. Cancer Lett. 2019;442::320–332.3039178210.1016/j.canlet.2018.10.015

The article "MicroRNA-744-5p suppresses tumorigenesis and metastasis of osteosarcoma through the p38 mitogen-activated protein kinases pathway by targeting transforming growth factor-beta 1" was retracted in 2026. Reasons: concerns about the data; concerns about the results or conclusions.

[29] Liang C, Xu J, Meng Q, et al. TGFB1-induced autophagy affects the pattern of pancreatic cancer progression in distinct ways depending on SMAD4 status. Autophagy. 2020;16(3):486–500.3117791110.1080/15548627.2019.1628540PMC6999639

[30] Loeffler I. MKP2 suppresses TGF-beta1-induced epithelial-to-mesenchymal transition through JNK inhibition. Clin Sci (Lond). 2019;133(3):545–550.3076064110.1042/CS20180881

[31] Dubash AD, Kam CY, Aguado BA, et al. Plakophilin-2 loss promotes TGF-beta1/p38 MAPK-dependent fibrotic gene expression in cardiomyocytes. J Cell Biol. 2016;212(4):425–438.2685826510.1083/jcb.201507018PMC4754716

[32] Sanchez-Capelo A. Dual role for TGF-beta1 in apoptosis. Cytokine Growth Factor Rev. 2005;16(1):15–34.1573383010.1016/j.cytogfr.2004.11.002

[33] Schiff L, Boles NC, Fernandes M, et al. P38 inhibition reverses TGFbeta1 and TNFalpha-induced contraction in a model of proliferative vitreoretinopathy. Commun Biol. 2019;2:162.3106927110.1038/s42003-019-0406-6PMC6499805

[34] Allen-Rhoades W, Kurenbekova L, Satterfield L, *et al*. Cross-species identification of a plasma microRNA signature for detection, therapeutic monitoring, and prognosis in osteosarcoma. Cancer Med. 2015;4(7):977–988.2578429010.1002/cam4.438PMC4529336

[35] Fleming JC, Woo J, Moutasim K, *et al*. CTEN induces tumour cell invasion and survival and is prognostic in radiotherapy-treated head and neck cancer. Cancers (Basel). 2020;12(10):2963.10.3390/cancers12102963PMC760210533066224

[36] Wang T, Zhang H, Wang H, et al. MiR-505-5p inhibits proliferation and promotes apoptosis of osteosarcoma cells via regulating RASSF8 expression. J BUON. 2021;26(2):599–605.34077011

[37] Ottaviani G, Jaffe N. The epidemiology of osteosarcoma. Cancer Treat Res. 2009;152:3–13.2021338310.1007/978-1-4419-0284-9_1

[38] Liu S, Wen C. miR-141-3p promotes retinoblastoma progression via inhibiting sushi domain-containing protein 2. Bioengineered. 2022;13(3):7410–7424.3525905110.1080/21655979.2022.2048770PMC8973658

[39] Wang Z, Sha HH, Li HJ. Functions and mechanisms of miR-186 in human cancer. Biomed Pharmacother. 2019;119:109428.3152564110.1016/j.biopha.2019.109428

[40] Yang X, Liu R. Long non-coding RNA HCG18 promotes gastric cancer progression by regulating miRNA-146a-5p/tumor necrosis factor receptor-associated factor 6 axis. Bioengineered. 2022;13(3):6781–6793.3524092010.1080/21655979.2022.2034565PMC8973972

[41] Ji Q, Xu X, Song Q, *et al*. miR-223-3p inhibits human osteosarcoma metastasis and progression by directly targeting CDH6. Mol Ther. 2018;26(5):1299–1312.2962830510.1016/j.ymthe.2018.03.009PMC5993963

The article "MicroRNA-744-5p suppresses tumorigenesis and metastasis of osteosarcoma through the p38 mitogen-activated protein kinases pathway by targeting transforming growth factor-beta 1" was retracted in 2026. Reasons: concerns about the data; concerns about the results or conclusions.

[42] Ma X, Li D, Gao Y, et al. miR-451a inhibits the growth and invasion of osteosarcoma via targeting TRIM66. Technol Cancer Res Treat. 2019;18:1533033819870209.3143454510.1177/1533033819870209PMC6706812

[43] Wang X, Peng L, Gong X, et al. miR-423-5p inhibits osteosarcoma proliferation and invasion through directly targeting STMN1. Cell Physiol Biochem. 2018;50(6):2249–2259.3042357610.1159/000495085

[44] Zhang W, Wei L, Sheng W, et al. miR-1225-5p functions as a tumor suppressor in osteosarcoma by targeting Sox9. DNA Cell Biol. 2020;39(1):78–91.3176522910.1089/dna.2019.5105

[45] Shen L, Wang P, Yang J, et al. MicroRNA-217 regulates WASF3 expression and suppresses tumor growth and metastasis in osteosarcoma. PLoS One. 2014;9(10):e109138.2528993610.1371/journal.pone.0109138PMC4188591

[46] Sun X, Dongol S, Qiu C, et al. miR-652 promotes tumor proliferation and metastasis by targeting RORA in endometrial cancer. Mol Cancer Res. 2018;16(12):1927–1939.3009356310.1158/1541-7786.MCR-18-0267

[47] De Craene B, Berx G. Regulatory networks defining EMT during cancer initiation and progression. Nat Rev Cancer. 2013;13(2):97–110.2334454210.1038/nrc3447

[48] Diepenbruck M, Christofori G. Epithelial-mesenchymal transition (EMT) and metastasis: yes, no, maybe? Curr Opin Cell Biol. 2016;43:7–13.2737178710.1016/j.ceb.2016.06.002

[49] Saitoh M. Involvement of partial EMT in cancer progression. J Biochem. 2018;164(4):257–264.2972695510.1093/jb/mvy047

[50] Jiang X, Zhang Z, Song C, et al. Glaucocalyxin A reverses EMT and TGF-beta1-induced EMT by inhibiting TGF-beta1/Smad2/3 signaling pathway in osteosarcoma. Chem Biol Interact. 2019;307:158–166.3105970610.1016/j.cbi.2019.05.005

[51] Odero-Marah V, Hawsawi O, Henderson V, et al. Epithelial-mesenchymal transition (EMT) and prostate cancer. Adv Exp Med Biol. 2018;1095:101–110.3022955110.1007/978-3-319-95693-0_6

[52] Suzuki HI, Kiyono K, Miyazono K. Regulation of autophagy by transforming growth factor-beta (TGF-beta) signaling. Autophagy. 2010;6(5):645–647.2045818410.4161/auto.6.5.12046

[53] Mishra AK, Parish CR, Wong ML, et al. Leptin signals via TGFB1 to promote metastatic potential and stemness in breast cancer. PLoS One. 2017;12(5):e0178454.2854257710.1371/journal.pone.0178454PMC5444832

[54] Song S, Qiu D, Luo F, et al. Knockdown of NLRP3 alleviates high glucose or TGFB1-induced EMT in human renal tubular cells. J Mol Endocrinol. 2018;61(3):101–113.3030716310.1530/JME-18-0069

[55] Gulubova M, Aleksandrova E, Vlaykova T. Promoter polymorphisms in TGFB1 and IL10 genes influence tumor dendritic cells infiltration, development and prognosis of colorectal cancer. J Gene Med. 2018;20(2–3):e3005.2938827710.1002/jgm.3005

The article "MicroRNA-744-5p suppresses tumorigenesis and metastasis of osteosarcoma through the p38 mitogen-activated protein kinases pathway by targeting transforming growth factor-beta 1" was retracted in 2026. Reasons: concerns about the data; concerns about the results or conclusions.

[56] Li T, Huang H, Shi G, et al. TGF-beta1-SOX9 axis-inducible COL10A1 promotes invasion and metastasis in gastric cancer via epithelial-to-mesenchymal transition. Cell Death Dis. 2018;9(9):849.3015445110.1038/s41419-018-0877-2PMC6113209

[57] Wu X, Zhao J, Ruan Y, et al. Sialyltransferase ST3GAL1 promotes cell migration, invasion, and TGF-beta1-induced EMT and confers paclitaxel resistance in ovarian cancer. Cell Death Dis. 2018;9(11):1102.3037537110.1038/s41419-018-1101-0PMC6207573

[58] Sharma S, Goswami R, Zhang DX, et al. TRPV4 regulates matrix stiffness and TGFbeta1-induced epithelial-mesenchymal transition. J Cell Mol Med. 2019;23(2):761–774.3045076710.1111/jcmm.13972PMC6349341

[59] Zhang X, Zhang P, Shao M, et al. SALL4 activates TGF-beta/SMAD signaling pathway to induce EMT and promote gastric cancer metastasis. Cancer Manag Res. 2018;10:4459–4470.3034937810.2147/CMAR.S177373PMC6188178

[60] Guan X, Zhao H, Niu J, et al. Polymorphisms of TGFB1 and VEGF genes and survival of patients with gastric cancer. J Exp Clin Cancer Res. 2009;28:94.1956694810.1186/1756-9966-28-94PMC2717936

[61] Juarez I, Gutierrez A, Vaquero-Yuste C, et al. TGFB1 polymorphisms and TGF-beta1 plasma levels identify gastric adenocarcinoma patients with lower survival rate and disseminated disease. J Cell Mol Med. 2021;25(2):774–783.3327479810.1111/jcmm.16131PMC7812301

[62] He J, Huang Z, He M, et al. Circular RNA MAPK4 (circ-MAPK4) inhibits cell apoptosis via MAPK signaling pathway by sponging miR-125a-3p in gliomas. Mol Cancer. 2020;19(1):17.3199230310.1186/s12943-019-1120-1PMC6986105

[63] Zhang L, Yang C, Huang Y, et al. Cardamonin inhibits the growth of human osteosarcoma cells through activating P38 and JNK signaling pathway. Biomed Pharmacother. 2021;134:111155.3337062810.1016/j.biopha.2020.111155

[64] Shi D, Wu F, Mu S, et al. LncRNA AFAP1-AS1 promotes tumorigenesis and epithelial-mesenchymal transition of osteosarcoma through RhoC/ROCK1/p38MAPK/Twist1 signaling pathway. J Exp Clin Cancer Res. 2019;38(1):375.3144366510.1186/s13046-019-1363-0PMC6708246

[65] Crimi S, Falzone L, Gattuso G, et al. Droplet digital PCR analysis of liquid biopsy samples unveils the diagnostic role of hsa-miR-133a-3p and hsa-miR-375-3p in oral cancer. Biology (Basel). 2020;9(11): 379.10.3390/biology9110379PMC769475033172167

[66] Mazumder S, Datta S, Ray JG, et al. Liquid biopsy: miRNA as a potential biomarker in oral cancer. Cancer Epidemiol. 2019;58:137–145.3057923810.1016/j.canep.2018.12.008

